# Longitudinal Association between Body Mass Index and Health-Related Quality of Life

**DOI:** 10.1371/journal.pone.0093071

**Published:** 2014-03-26

**Authors:** Jacqueline Müller-Nordhorn, Rebecca Muckelbauer, Heike Englert, Ulrike Grittner, Hendrike Berger, Frank Sonntag, Heinz Völler, Christof Prugger, Karl Wegscheider, Hugo A. Katus, Stefan N. Willich

**Affiliations:** 1 Institute for Social Medicine, Epidemiology and Health Economics, Charité – Universitätsmedizin Berlin, Berlin, Germany; 2 Berlin School of Public Health, Charité – Universitätsmedizin Berlin, Berlin, Germany; 3 University of Applied Sciences, Münster, Germany; 4 Department of Biostatistics and Clinical Epidemiology, Charité – Universitätsmedizin Berlin, Berlin, Germany; 5 University of Applied Sciences, Osnabrück, Germany; 6 Cardiology Practice, Henstedt-Ulzburg, Germany; 7 Centre of Rehabilitation Research, University of Potsdam, Potsdam, Germany; 8 Paris Cardiovascular Research Centre, University Paris Descartes, Sorbonne Paris Cité, UMR-S970, Paris, France; 9 Department of Medical Biometry and Epidemiology, University of Hamburg, Hamburg, Germany; 10 Department of Cardiology, Angiology and Pneumology, University of Heidelberg, Heidelberg, Germany; Pennington Biomedical Research Center, United States of America

## Abstract

**Objective:**

Health-related quality of life (HRQoL) is an important outcome in individuals with a high risk for cardiovascular diseases. We investigated the association of HRQoL and body mass index (BMI) as an indicator for obesity.

**Design:**

Secondary longitudinal analysis of the ORBITAL study, an intervention study which included high-risk cardiovascular primary care patients with hypercholesterolemia and an indication for statin therapy.

**Methods:**

HRQoL was determined with the generic Short Form (SF)-12 health status instrument. Body weight and height were assessed at baseline and at months 6, 12, 18, 24, 30, and 36. We used a linear and a linear mixed-effects regression model to investigate the association between BMI and SF-12 summary scores at baseline as well as between change in BMI and SF-12 summary scores over 3 years. We adjusted for age, sex, smoking status, and in the longitudinal analysis also for the study arm and its interaction term with time.

**Results:**

Of the 7640 participants who completed the baseline questionnaire, 6726 participants (mean age: 61 years) were analyzed. The baseline BMI was inversely associated with physical and mental SF-12 summary scores (β [95% CI] per 1 kg/m^2^: −0.36 [−0.41; −0.30] and −0.05 [−0.11; −0.00], respectively). A significant association between the change in BMI and physical SF-12 summary scores over time was only present in women (−0.18 [−0.27; −0.09]) and only in obese participants (−0.19 [−0.29; −0.10]). A change in BMI was directly associated with mental SF-12 summary scores (0.12 [0.06; 0.19]) in the total population.

**Conclusion:**

Increases in BMI were associated with decreases in physical HRQoL, particularly in obese individuals and in women. In contrast, the mental HRQoL seemed to increase with increasing BMI over time. Thus, body weight management with respect to the HRQoL should be evaluated differentially by sex and body weight status.

**Trial Registration:**

ClinicalTrials.gov NCT00379249

## Introduction

The obesity epidemic is a major public health challenge in an increasing number of countries worldwide [1]. For the individual, the major consequences of obesity include an increased risk of both all-cause and, in particular, cardiovascular mortality [2]–[4]. In addition, obesity is a risk factor for several morbidities, such as type 2 diabetes mellitus [5], [6], and it is associated with psychological disorders, such as depression, and social discrimination [5]–[7].

Obesity is also an important indicator for health-related quality of life (HRQoL) [8]–[37]. HRQoL, which can be classified into physical and mental components, is both a predictor for future health status and an outcome itself. It has been shown to predict premature mortality [38]–[43] and morbidities such as type 2 diabetes mellitus and cardiovascular events [42], [44], [45]. HRQoL as an outcome is especially relevant for individuals with chronic diseases who spend an increasing amount of time living with their disease due to improved survival.

The cross-sectional association between measures of obesity and HRQoL in various populations has been broadly studied [8]–[31], [37]. In most studies, HRQoL was reduced in underweight and obese individuals; typically it was highest for individuals with a body mass index (BMI) between around 18.5 kg/m^2^ and 25 kg/m^2^, i.e., normal-weight individuals [8]–[15], [24], [26].

In contrast, only a few studies have investigated the longitudinal association between measures of obesity and HRQoL. In populations with diabetes or hypertension, a higher BMI was a predictor for later decreased physical HRQoL but not for mental HRQoL [32], [33]. Three cohort studies indicated that weight gain over time was linked to an impairment of physical HRQoL [34]–[36]. With the exception of these results, there is a lack of evidence that a change in body weight has an impact on later HRQoL.

In the present study, we analyzed data from patients with a high risk for cardiovascular diseases. We investigated the longitudinal impact of a change in BMI on HRQoL over a 3-year study period. In addition, we analyzed the cross-sectional association between baseline BMI and HRQoL.

## Materials and Methods

### Study Design

The analyzed patient cohort originated from the ORBITAL (Open Label Primary Care Study: Rosuvastatin Based Compliance Initiatives to Achievements of LDL Goals) study. This study was a randomized controlled trial, registered at www.clinicaltrials.gov with the identifier NCT00379249. The design and results are described in detail elsewhere [46], [47]. The primary aim of this intervention study was to investigate the cost-effectiveness of an adherence-enhancing intervention in patients with hypercholesterolemia at primary care practices. Participants were randomized to receive rosuvastatin therapy alone or together with an adherence program for 1 year, followed by a 2-year observational period. In a secondary longitudinal analysis of this intervention study combining all participant data, we investigated the association between BMI and HRQoL measured at baseline and at six follow-up points within 3 years.

### Ethics Statement

The ethics committee of the Charité – Universitätsmedizin Berlin approved the study protocol. All of the participants gave written informed consent before study inclusion.

### Study Population

In the ORBITAL study, the participants were enrolled with hypercholesterolemia and an indication for statin therapy from 1961 primary care practices in Germany. The participants had to have low-density lipoprotein cholesterol levels ≥3.0 mmol/l for drug-naïve individuals or ≥3.25 mmol/l for participants who were already on lipid-lowering therapy and with at least one of the following risk factors: diabetes, a history of coronary heart disease or other atherosclerotic disease, or an absolute coronary heart disease risk ≥20% over 10 years according to the Framingham criteria [48].

For the present analyses, we included all of the participants of the ORBITAL study with an available baseline questionnaire. We excluded participants with missing baseline data and those without paired data on BMI, HRQoL, and smoking status for at least one follow-up point. In addition, we excluded participants who were underweight, defined as a BMI <18.5 kg/m^2^. The size of the subsample of underweight individuals (n = 50) was too small to allow subgroup analyses by BMI category. Also, underweight is often associated with underlying diseases and an increased mortality, especially in the elderly, even after controlling for cancer and cardiovascular diseases [49], [50]. The impact of these diseases on HRQoL and weight-changes is difficult to disentangle and may introduce confounding by indication.

### Assessments and Included Variables

At baseline, the participants filled out a standardized self-administered questionnaire. Physicians assessed the participants’ medical history and performed a physical examination. The follow-up data were collected from the participants by postal questionnaires every 6 months during a period of 3 years at the 6-, 12-, 18-, 24-, 30-, and 36-month follow-up points. In addition, a physical examination was performed at the 6- and 12-month follow-up points.

#### Health-related quality of life (HRQoL)

HRQoL was assessed at baseline and at all of the follow-up points with the standard 4-week recall version 1 of the Short Form-12 (SF-12), a generic health status instrument [51]. The SF-12 includes one or two items from each of the eight health concepts of the instrument SF-36 [51]. The SF-12 allows the calculation of the physical and mental component summary scores. The items selected for the SF-12 summary scales and the scoring algorithms were cross-validated in nine countries [52]. The SF-12 summary scales were calculated directly from the 12 items and were set missing if the respondent was missing any one of the items. Higher physical or mental SF-12 summary scores indicated a better HRQoL.

#### BMI, BMI categories, and weight-change groups

The body weight and height were assessed to the nearest kilogram and centimeter, respectively. They were self-reported by the participants in the baseline questionnaire and in the six follow-up questionnaires. In addition, physicians assessed body weight and height at baseline and at the 6- and 12- month follow-up. We calculated the BMI by dividing the self-reported body weight in kilograms by the baseline physician-reported height in meters squared (kg/m^2^). In the case of missing data for physician-reported height, the self-reported height at baseline was used. We used self-reported body weight to calculate the BMI allowing for consistency across all assessment points. We applied the World Health Organization (WHO) classification to categorize BMI values into the following BMI categories: underweight (BMI<18.5 kg/m^2^), normal weight (BMI 18.5 to <25 kg/m^2^), overweight (BMI 25 to <30 kg/m^2^), and obese (≥30 kg/m^2^) [5]. To differentiate between individuals with weight gain, stable weight, and weight loss from baseline to the 36-month follow-up, we classified the study population into three weight-change groups: weight loser (BMI change within 36 months <**−**0.5 kg/m^2^), stable weight (BMI change **−**0.5 to 0.5 kg/m^2^), and weight gainer (BMI change >0.5 kg/m^2^). These BMI change cut-offs were based on the cut-offs used in a comparable study on weight-change groups [35].

#### Smoking status and other covariates

We assessed socio-demographic variables such as age, sex, education level, living situation, and employment status by using standardized self-administered questionnaires at baseline. The living situation indicated whether the participants lived alone or not. Participants were categorized by their employment status according to whether they currently worked in a job or not. The education level was categorized into three levels according to the number of school years needed for the different levels of school graduation: low (≤9 years), middle (10 years), and high (12 to 13 years). Participants’ smoking status was categorized into three categories: current, former, and never smoker. The medical history was assessed at baseline and included diagnosis of diabetes and hypertension, history of myocardial infarction and stroke, as well as history of coronary artery bypass graft (CABG) and percutaneous coronary intervention (PCI) procedures. For each diagnosis or procedure, a binary variable was built. Cardiovascular events and revascularization procedures during follow-up were self-reported by participants in the questionnaires at the six follow-up points. A time-dependent variable, cumulative incidence of myocardial infarction or stroke, was generated by cumulating a dummy variable for the incidence of at least one of these events during the previous 6 months at each follow-up point. The time-dependent variable, cumulative incidence of CABG or PCI, was generated in the same way.

### Statistical Analyses

First, we analyzed the relative validity of the BMI that we calculated using the self-reported body weight (hence: self-reported BMI) by comparing it with the BMI calculated using the physician-reported body weight (hence: physician-reported BMI). For the validation analysis, we used all of the available data from the ORBITAL study population at baseline. We calculated the Spearman correlation coefficient to determine the correlation between the self-reported and physician-reported BMI. To identify systematic and BMI-dependent differences between the two assessment methods, we used the Bland-Altman plot [53]. The difference between self-reported and physician-reported BMI was plotted against the average of both. The limits of agreement were defined by the mean difference ±2 standard deviations (SD) as suggested by Bland and Altman [53]. The association of the difference between the two assessment methods with the average of the two methods was tested by regression analysis. We also performed regression analyses to test for an association of the difference between the two assessment methods with the two SF-12 summary scores.

We performed descriptive statistical analysis for the baseline characteristics of the analyzed study population and stratified by BMI category and weight-change group. Baseline SF-12 summary scores were also provided for three age groups (<40 years, 40 to <60 years, and ≥60 years). The arithmetic means (±SD) or percentages were reported.

The cross-sectional association between the baseline BMI and baseline SF-12 summary scores was estimated using a linear regression model, which was adjusted for age, sex, and smoking status at baseline. We adjusted for smoking status as a potential confounder due to its association with both BMI and HRQoL in previous studies [11], [14], [32], [33]. In a further adjusted model, we additionally controlled for the potential confounders: education level, employment status, living situation, diagnosis of diabetes and hypertension, history of myocardial infarction, stroke, and CABG and PCI procedures at baseline.

The longitudinal association between change in BMI and SF-12 summary scores over the 3-year study period was estimated by using a linear mixed-effects regression model (PROC MIXED in SAS 9.3). The physical and mental SF-12 summary scores at baseline and at the six follow-up points were defined as the dependent variables in separate models. The models included the following as independent variables: change in BMI (as a time-dependent variable), baseline BMI, and time (as a categorical variable with seven levels: baseline and six follow-up points). The change in BMI was calculated at each follow-up point by subtracting the BMI value at baseline from the BMI value at the respective follow-up point. The regression coefficients (β) for change in BMI (in kg/m^2^) were generated in a linear mixed-effects regression model. These models have the advantage to deal with missing values because they use all of the available data from an individual during follow-up. A random statement was included to account for the initial differences between individuals. A repeated statement with a heterogeneous autoregressive covariance structure fitted best (according to Akaike’s information criterion) to account for correlations on the individual level between the repeated measures at baseline and the six follow-up points. This basic model was controlled for age, sex, and smoking status (as a time-dependent variable). Since we analyzed data from an intervention study, we also adjusted the basic model for the study arm (two levels: intervention and control group) and the interaction term time × study arm. A further adjusted model additionally controlled for the education level, employment status, living situation, diagnosis of diabetes and hypertension, history of myocardial infarction, stroke, and CABG and PCI procedures at baseline, with the combined cumulative incidence of myocardial infarction or stroke and the combined cumulative incidence of CABG or PCI procedures within the previous 6 months as time-dependent variables. The random effects parameters of the mixed-effects models are reported for the basic models.

To investigate the possible effect modifications with sex and baseline BMI category, the interaction terms with baseline BMI and change in BMI were separately entered into the basic models of the cross-sectional and longitudinal analyses. In the case of a significant interaction term, post-hoc subgroup analyses were performed and regression coefficients are presented.

All of the tests for significance were two-sided; the significance level was α = 0.05. The statistical analyses were performed using SAS 9.3 (SAS Institute Inc., Cary, North Carolina, US) and the figures were created with SPSS 19 (SPSS Inc., Chicago, Illinois, US). No adjustment for multiple testing was applied.

## Results

### Study Population

**Figure 1** shows the participant flow from randomization in the ORBITAL study to the combined study population included in our analyses. At baseline, 7640 participants completed the self-administered questionnaire. We analyzed 6726 participants in the basic models. In the further adjusted models, 6682 participants could be analyzed because of the missing values of the additional variables. In **Table 1**, the baseline characteristics including the SF-12 summary scores of the analyzed study population are presented, which are also stratified by BMI category. At baseline, the mean (±SD) physical SF-12 summary score was 49.7±8.1 in the age group of <40 years, 45.5±10.2 in the age group of 40 to <60 years, and 44.2±9.9 in participants aged ≥60 years. The respective means of the mental SF-12 summary score were 50.6±9.4, 50.4±9.8, and 44.2±9.9.

**Figure 1:** Participant flow from randomization in the ORBITAL intervention study to analyses of the present study. Abbreviations: BMI = body mass index, CABG = coronary artery bypass graft, HRQoL = health-related quality of life, ORBITAL = Open Label Primary Care Study Rosuvastatin Based Compliance Initiatives to Achievements of LDL Goals, PCI = percutaneous coronary intervention.

**Table 1:** Baseline characteristics and SF-12 summary scores of the analyzed study population, stratified by BMI category.

Variables^1^	Totalpopulation	Normal weight (BMI 18.5to <25 kg/m^2^)	Overweight (BMI 25to <30 kg/m^2^)	Obese (BMI≥30 kg/m^2^)
No.	6726	1493	3288	1945
Physical SF-12 summary score (mean±SD)^2^	45±10	46±10	45±10	43±10
Mental SF-12 summary score (mean±SD)^2^	52±9	52±9	52±9	52±10
Age (years, mean±SD)	61*±*10	61*±*11	61±10	60±10
Male (%)	57	51	63	51
Intervention group (%)	50	51	50	49
Body mass index (kg/m^2^, mean±SD)	28*±*4	23±1	27±1	33±3
LDL cholesterol (mg/dl, mean±SD)	170*±*39	173±40	171±39	168±38
Education level (%)^3^				
Low (≤9 school years)	64	58	64	68
Middle (10 school years)	19	21	19	18
High (12 to 13 school years)	17	21	16	13
Living alone (%)	19	21	17	20
Actively employed (%)	33	34	33	31
Smoking status (%)				
Current smoker	21	27	21	18
Former smoker	36	27	39	38
Never smoker	43	46	40	45
Hypertension (%)	58	46	56	71
Diabetes (%)	28	17	25	43
History of myocardial infarction (%)	16	14	19	14
History of stroke (%)	7	6	7	7
History of coronary artery bypass graft (%)	10	9	12	7
History of percutaneous coronaryintervention (%)	12	10	13	10

Abbreviations: LDL = low-density lipoprotein, SD = standard deviation, SF = Short Form.

1 Percentages may not add up due to rounding.

2 Score could range between 0 and 100 and was assessed with the SF-12 health status instrument.

3 Categorization by the number of school years needed for the different levels of school graduation.

### Relative Validity of Self-reported BMI

The paired data for the validation of BMI calculated with the self-reported body weight against the physician-reported body weight was available for 7570 participants. The Spearman correlation coefficient for the correlation between the self-reported and physician-reported BMI was r = 0.976 demonstrating a nearly perfect linear relationship between both of the measures. The Bland-Altman analysis indicated that BMI was underestimated on average by **−**0.1 kg/m^2^ when calculated with self-reported body weight (**Figure 2**). The limits of agreement between the two assessment methods ranged from **−**1.9 to 1.7 kg/m^2^. The visual analysis of the plot and the results of the regression analysis (β = **−**0.003, P = 0.190) did not suggest that the difference between the two assessment methods depended on the participants’ BMI, which was calculated as the average of the two assessment methods. Similarly, the difference in BMI measured by the two methods was not associated with the self-reported physical and mental SF-12 summary scores (β = 0.001, P = 0.718 and β = 0.001, P = 0.350, respectively).

**Figure 2:** Bland Altman plot for baseline BMI calculated from the self-reported and physician-reported body weight. The bias (mean) between the two methods is marked by the full line (–), the upper and lower limits of agreement (mean ±2 standard deviations) by the dotted line (···) and the regression line by the broken line (− − −). Six observations are outside the axis range. Abbreviation: BMI = body mass index.

### Cross-sectional Association between BMI and HRQoL

#### Physical SF-12 summary score

On the cross-sectional level, BMI was inversely associated with physical SF-12 summary scores in the basic model, adjusted for age, sex, and smoking status, i.e., physical SF-12 summary scores decreased with increasing BMI (**Table 2**). The further adjusted model confirmed this association controlling for education level, employment status, living situation, diagnosis of diabetes and hypertension, and history of myocardial infarction, stroke, and CABG and PCI procedures. There was a significant interaction in the basic model between baseline BMI category and baseline BMI with regard to physical SF-12 scores. In overweight and obese participants, BMI (in kg/m^2^) was inversely associated with physical SF-12 summary scores (β: **−**0.47, P<0.001 and β: **−**0.42, P<0.001, respectively). In contrast, in normal-weight participants, BMI was not significantly associated with physical SF-12 summary scores (β: 0.33, P = 0.082). There was no significant interaction between sex and baseline BMI (**Table 2**).

**Table 2:** Cross-sectional association of baseline BMI with the mental and physical SF-12 summary scores, stratified by BMI category.

	Population	Association betweenbaseline BMIand SF-12 summaryscore^1^			Interaction ofbaseline BMIwith sex	Interaction ofbaseline BMIwith baselineBMI category
		β^2^	[95% CI]	P	P	P
**Physical SF-12 summary score**						
Basic model^3^	total	−0.36	[−0.41; −0.30]	<0.001	0.227	0.003
Further adjusted model^4^	total	−0.35	[−0.37; −0.32]	<0.001		
Post-hoc analysis by baselineBMI category^3^^,^ 5	normalweight	0.33	[−0.04; 0.70]	0.082		
	overweight	−0.47	[−0.71; −0.23]	<0.001		
	obese	−0.42	[−0.57; −0.28]	<0.001		
**Mental SF-12 summary score**						
Basic model^3^	total	−0.05	[−0.11; −0.00]	0.045	0.976	0.488
Further adjusted model^4^	total	−0.05	[−0.07; −0.03]	<0.001		

Abbreviations: BMI = body mass index, CI = confidence intervals, SF = Short Form.

1 Stratified regression coefficients are reported only with significant interaction terms in the basic model (P<0.05).

2 β can be interpreted as difference in SF-12 summary score per increase in baseline BMI of 1 kg/m^2^.

3 Basic model included the SF-12 summary score at baseline as the dependent variable and baseline BMI, age, sex, and smoking status at baseline as independent variables, n = 6726.

4 Further adjusted model consisting of the basic model additionally adjusted for education level, employment status, living situation, diagnosis of diabetes and hypertension, and history of myocardial infarction, stroke, coronary artery bypass grafting, and percutaneous coronary intervention at baseline, n = 6682.

5 Normal weight (BMI 18.5 to <25 kg/m^2^), overweight (BMI 25 to <30 kg/m^2^), and obese (BMI ≥30 kg/m^2^).

#### Mental SF-12 summary score

There was a significant albeit small inverse cross-sectional association between BMI and mental SF-12 summary score (β: **−**0.05, P = 0.045) in the basic model (**Table 2** **)**. The association remained after further adjustment for education level, employment status, living situation, diagnosis of diabetes and hypertension, and history of myocardial infarction, stroke, and CABG and PCI procedures. The interactions of baseline BMI with baseline BMI category and with sex were not significant (**Table 2**).

### Longitudinal Association between BMI and HRQoL

**Figure 3** shows the mean changes in physical and mental SF-12 summary scores from baseline to the 36-month follow-up according to baseline BMI category in the three weight-change groups. The mean change (±SD) in BMI during the 36-month follow-up was 0.1±1.7 kg/m^2^.

**Figure 3:** Mean changes in the physical (part A) and mental (part B) SF-12 summary scores from baseline to 36-month follow-up according to baseline BMI category in three weight-change groups. Weight-change groups: weight loser (BMI change over 36 months <−0.5 kg/m^2^), stable weight (BMI change −0.5 to 0.5 kg/m^2^), and weight gainer (BMI change >0.5 kg/m^2^). Abbreviations: BMI = body mass index in kg/m^2^, SF = Short Form.

#### Physical SF-12 summary score

The mixed-effects model revealed a significant inverse association between change in BMI and physical SF-12 summary scores over time, adjusted for baseline BMI, age, sex, smoking status, study arm, and the interaction term time × study arm (**Table 3**). The association remained significant after further adjustment for education level, employment status, living situation, diagnosis of diabetes and hypertension, and history and time-dependent cumulative incidence of myocardial infarction/stroke and CABG/PCI. There were significant interactions between change in BMI with baseline BMI category and with sex. In initially obese participants, an increase in BMI was associated with a reduction in physical SF-12 summary scores over time (β: **−**0.19, P<0.001), whereas there was no association in normal-weight and overweight participants (**Table 3**). Stratified analysis by sex showed that the inverse association between change in BMI and physical SF-12 summary scores over time was significant only in women (β: **−**0.18, P<0.001) (**Table 3**).

**Table 3:** Longitudinal association of change in BMI with the mental and physical SF-12 summary scores during the 3-year follow-up, stratified by sex and BMI category.

	Population	Association between changein BMI and SF-12 summaryscore during follow-up^1^			Interaction of changein BMIwith sex	Interaction of changein BMI withbaseline BMIcategory
		β^2^	[95% CI]	P	P	P
**Physical SF-12** **summary score**						
Basic model^3^	total	−0.09	[−0.15; −0.03]	0.004	0.015	0.033
Further adjusted model^4^	total	−0.09	[−0.16; −0.03]	0.003		
Post-hoc analysis by sex^3^	women	−0.18	[−0.27; −0.09]	<0.001		
	men	−0.01	[−0.09; −0.07]	0.821		
Post-hoc analysis by baselineBMI category^3^^,^ 5	normalweight	0.00	[−0.15; 0.16]	0.959		
	overweight	−0.02	[−0.12; 0.07]	0.632		
	obese	−0.19	[−0.29; −0.10]	<0.001		
**Mental SF-12 summary** **score**						
Basic model^3^	total	0.12	[0.06; 0.19]	<0.001	0.484	0.089
Further adjusted model^4^	total	0.13	[0.06; 0.19]	<0.001		

Abbreviations: BMI = body mass index, CI = confidence intervals, SF = Short Form.

1 Stratified regression coefficients are reported only in the case of significant interaction terms in the basic model (P<0.05).

2 β can be interpreted as the change in SF-12 summary score per increase in BMI change of 1 kg/m^2^ over time.

3 Basic model included the SF-12 summary score at all time points as the dependent variable and baseline BMI, change in BMI from baseline to all follow-up points, age, sex, study arm, interaction term time × study arm, and time-dependent smoking status as independent variables, n = 6726.

4 Further adjusted model consisting of the basic model additionally adjusted for education level, employment status, living situation, diagnosis of diabetes and hypertension, and history and time-dependent cumulative incidence of myocardial infarction/stroke and coronary artery bypass grafting/percutaneous coronary intervention within the previous 6 months, n = 6682.

5 Normal weight (BMI 18.5 to <25 kg/m^2^), overweight (BMI 25 to <30 kg/m^2^), and obese (BMI ≥30 kg/m^2^).

As estimated in the basic mixed-effects model, the variance in baseline physical SF-12 summary score between individuals (random effects parameter for the intercept) was 66.1 (standard error [SE]: 1.3). The variance between the individuals by the seven time points (random effects for the different time points) ranged from 27.4 (SE: 0.6) at the 12-month follow-up to 41.3 (SE: 0.8) at the 36-month follow-up. The heterogeneous autoregressive variance parameter was 0.20 (SE: 0.01).

#### Mental SF-12 summary score

With regard to the mental SF-12 summary score, an increase in BMI by 1 kg/m^2^ was associated with a higher mental SF-12 summary score by 0.12 score units (P<0.001) in the basic model (**Table 3**). The association was similar after further adjustment for education level, employment status, living situation, diagnosis of diabetes and hypertension, and history and time-dependent cumulative incidence of myocardial infarction/stroke and CABG/PCI. There was no significant interaction between change in BMI and baseline BMI category or sex (**Table 3**).

The random effects parameter for the baseline mental SF-12 summary score was 52.6 (SE: 1.1). The random effects for the different time points ranged from 30.7 (SE: 0.7) at the 12-month follow-up to 47.6 (SE: 0.7) at the 36-month follow-up. The heterogeneous autoregressive variance parameter was 0.15 (SE: 0.01).

## Discussion

In the present study, we investigated the cross-sectional and the longitudinal association between BMI and HRQoL over 3 years in individuals with a high risk for cardiovascular diseases. In the cross-sectional analyses, BMI was inversely associated with physical and mental HRQoL, measured by the SF-12 health status instrument. The longitudinal analyses showed that change in BMI was inversely related to physical HRQoL in women and in obese individuals. In contrast, change in BMI was directly associated with mental HRQoL over time.

### Cross-sectional Association between BMI and HRQoL

Numerous cross-sectional studies have affirmed that compared to normal-weight individuals, obese individuals are more likely to have a poorer level of physical HRQoL [8]–[17], [22], [25], [30], [31], [34], [37]. Our study results confirmed that BMI is inversely associated with physical SF-12 summary score. In addition, the cross-sectional association seemed to be non-linear. In overweight and obese individuals, the physical SF-12 summary score decreased with increasing BMI whereas no such association was found in normal-weight individuals. Several studies identified the highest levels of physical HRQoL among normal-weight adults [8]–[11], [13], [16], [17], [30], [54]. However, other studies showed significantly poorer physical HRQoL only in obese but not in overweight individuals [14], [15], [31], [37]. Studies that modeled a non-linear relationship identified different peak values of physical HRQoL at BMI-ranges from <20 to about 30 kg/m^2^ [10], [26], [29], [54].

The literature is less consistent in reporting an association between BMI and mental HRQoL. In several studies, obesity was related to the physical but not to the mental HRQoL components [11]–[13], [16]–[18], [22], [34], [37], [54]. Other studies showed an association between obesity and the mental HRQoL [8], [10], [14], [26], [31], [55], whereas the association was often much weaker compared to the physical components [11], [12], [16]. Our study confirmed a weak but significant inverse cross-sectional relationship between BMI and mental HRQoL. Several studies indicated a non-linear association between BMI and mental HRQoL [8], [10], [12], [26], [54]. According to our data, there was no significant interaction between baseline BMI and BMI category, which did not hint at a non-linear association between BMI and mental SF-12 summary score.

### Longitudinal Association between Changes in BMI and HRQoL

Weight gain, indicated by an increase in BMI, was associated with decreased physical HRQoL over time in women and in obese individuals. Up to now, only a few studies have investigated the longitudinal association between change in body weight measures and HRQoL over time [34]–[36]. Cameron *et al.* showed in a population-based study in Australia that weight gain over 5 years was associated with an impaired physical HRQoL as measured by the SF-36 questionnaire [34]. Similar to our results, this negative impact of additional weight gain over time was greatest in the obese participants and tended to be stronger in women compared to men. This difference by gender was also observed in a British cohort study with middle-aged adults that combined retrospective and prospective assessments of body weight with a median follow-up time of 49 years [36]. Women, but not men, in the highest average weight gain tertile were more likely to have poor physical functioning compared to their counterparts in the lowest tertile [36]. Fine *et al.* analyzed the association of weight loss and weight gain over 4 years with HRQoL in middle- to older-aged women of the Nurses’ Health Study [35]. In this study, weight gain was associated with a decreased physical function score in all age and BMI groups. Weight loss, on the other hand, was associated with a slight improvement in physical HRQoL among overweight and obese women [35]. The descriptive analysis of our data also indicated that compared to weight loss, weight gain is more strongly associated with a decrease in physical HRQoL in obese individuals. To conclude, there seems to be an adverse impact of weight gain on physical HRQoL, especially in obese individuals and in women.

Our analyses showed that the mental SF-12 summary score was directly associated with BMI over time. The descriptive analysis indicated that weight loss, rather than weight gain, was associated with a decrease in mental HRQoL, especially among normal-weight individuals. Such an association was also reported by Fine *et al.* in the Nurses’ Health Study [35]. They found that losing 2 to 9 kg of body weight was associated with a decrease in the mental HRQoL, especially in women ≥65 years of age [35]. On the other hand, weight gain >9 kg was also associated with a reduction in the mental health score, but only in overweight and obese women. The study by Cameron *et al.* did not find any association between change in body weight over 5 years and mental HRQoL [34].

Explanations for the decreasing mental HRQoL with decreasing BMI remain speculative. Fine *et al.* suggested unintentional weight loss as a reason for the association in women in the Nurses’ Health Study [35]. Unintentional weight loss can be a symptom of an underlying disease such as undiagnosed cancer and psychiatric problems that may also have an impact on HRQoL [56]. A disease that was shown to be more strongly correlated with the mental rather than the physical HRQoL is depression [57]. Because depression is considered to be a main cause of unintentional weight loss in the elderly [58], it could be an underlying disease causing weight loss and reduced mental HRQoL.

#### Limitations

A major limitation of the present analyses is that BMI and HRQoL were self-reported which may introduce measurement bias. Thus, we validated self-reported BMI with physician-reported BMI. The results indicated that underreporting by participants was on average very low. Because the difference between the two measurement methods neither depended on the baseline BMI nor on the SF-12 summary scores, our data does not support a differential measurement bias by these factors. However, calculated changes in BMI over time may be imprecise because of the high individual imprecision of the self-reported BMI. This may reduce the power to show differences in HRQoL associated with changes in BMI.

Our study population consisted of primary care patients with hypercholesterolemia and an indication for statin therapy, and thus is not representative for the general population. However, the age-specific physical and mental SF-12 summary scores were similar to the German general population in the age group of ≥60 years, whereas in the younger age groups (<40 years and 40 to <60 years) both summary scores were slightly lower [59].

Another limitation is the linear modeling of the associations between BMI and HRQoL. To detect a possible non-linearity, we tested for an interaction of baseline BMI with BMI category and, in consequence, stratified the analyses. Our results suggest non-linear associations between BMI and physical HRQoL. To facilitate the interpretation of the results, we had decided to use the BMI categories according to the WHO classification. Other models without BMI categorization may result in a better model fit.

A strength of our longitudinal analysis was the application of the mixed-effects model which used all available data of the baseline and the six follow-up points by multilevel modeling. This method also considered individuals with missing data at some follow-up points. Thus, selection bias by the exclusion of participants with missing data could be reduced.

### Clinical Relevance

We found a significant longitudinal association between BMI and physical HRQoL. With each increase in BMI due to weight gain the physical SF-12 summary score decreased over time in the overall study population. Stratified analysis revealed that this inverse association was definite in obese individuals and in women. In obese participants, for example, each increase in BMI by 1 kg/m^2^ was associated with a decreased physical SF-12 summary score by 0.19 units over 3 years. The clinical relevance of the observed association may thus be limited during the 3-year follow-up period. However, considering weight gain over the lifespan the clinical relevance might increase over the long term.

A beneficial impact of weight change would become relevant if population groups are identified for which interventions for weight loss or weight maintenance have the potential to increase or maintain HRQoL. Maciejewski *et al*. found in their review and meta-analysis that interventions for weight loss can improve HRQoL but study results were inconsistent [54]. In weight-loss interventions, it can be difficult to distinguish between the effect of the reduced body weight on HRQoL and the effect of the components of the program such as increased physical activity or improved diet. Two studies investigating this difference showed that the individual’s weight loss could not completely but partly explain the beneficial intervention effect on physical HRQoL [55], [56].

We observed that weight gain was associated with a decrease in physical HRQoL in women but not in men. This result was in accordance with two of the three longitudinal studies [34], [36] in which the impact of weight gain on physical HRQoL was more pronounced in women compared to men. The third longitudinal study included only women [35]. Maciejewski *et al.* could not analyze the effect of weight loss interventions on HRQoL in their meta-analysis for the subgroup of women [60]. Statistical pooling of the data was not possible as the original data was unavailable to the authors. Thus, weight loss interventions may be especially appropriate in the target group of obese women but more research is needed to investigate gender differences in the association between BMI and HRQoL.

## Conclusion

Physical HRQoL decreases with increasing BMI in overweight and obese individuals. Mental HRQoL seems to be slightly poorer in individuals with a higher BMI. Weight gain over time was associated with an impairment of the physical HRQoL. In contrast, weight loss seems to result in a reduced mental HRQoL. The negative impact of weight gain on the physical HRQoL seems to be specifically relevant in obese individuals and in women, and these could be target groups for preventive and therapeutic interventions that aim at improved HRQoL. An adverse effect of weight loss on mental HRQoL over time needs to be replicated in further studies considering factors such as unintentional weight loss.
